# Gynostemma Glycosides Protect Retinal Ganglion Cells in Rats with Chronic High Intraocular Pressure by Regulating the STAT3/JAK2 Signaling Pathway and Inhibiting Astrocyte and Microglia Activation

**DOI:** 10.1155/2022/9963754

**Published:** 2022-08-11

**Authors:** Xian-jing Wang, Rong Hu, Qiong-ying Huang, Qing-hua Peng, Juan Yu

**Affiliations:** ^1^Hunan University of Chinese Medicine, Changsha, China; ^2^Hunan Provincial Key Laboratory for the Prevention and Treatment of Ophthalmology and Otolaryngology Diseases with Traditional Chinese Medicine, Changsha, China; ^3^The First Affiliated Hospital, Hunan University of Chinese Medicine, Changsha, China

## Abstract

**Objective:**

To observe the protective effect of gynostemma glycosides on retinal ganglion cells in rats with chronically high intraocular pressure.

**Materials and Methods:**

A total of 60 rats were randomly divided into group A (the blank group, 10 rats) and chronic high IOP model group (50 rats). The IOP model group (IOP above 22 mmHg) was then randomly divided into an additional 5 groups (10 rats per group): group B (negative control group) treated with normal saline; group C treated with gynostemma glycosides 25 mg/(kg-d); group D treated with gynostemma glycosides 50 mg/(kg-d); group E treated with gynostemma glycosides 100 mg/(kg-d); and group F (positive control group) treated with VitB1 and VitB12. The eyes of each rat were monitored from day 1 to 14 (D1–D14). On day 14, rats were euthanized, after which retinal tissue and optic nerve were examined using real-time PCR, western blot, HE staining, LFB staining, and TUNEL assay.

**Results:**

Groups A, C, D, E, and F had significantly lower expression of CD11b, GFAP, Brn3*α*, and more TUNEL cells than in group B (all *P* < 0.05). Moreover, the relative expression of STAT3 mRNA and JAK2 (mRNA and protein) in groups A, C, D, E, and F was significantly lower than in group B (*P* < 0.05), while in group E, the expression was lower than in group D (*P* < 0.05).

**Conclusion:**

Gynostemma glycosides protect retinal ganglion cells in rats with chronically high intraocular pressure possibly associated with the STAT3/JAK2 signaling pathway.

## 1. Introduction

Glaucoma is a disease characterized by optic nerve atrophy and visual field defects and is the leading cause of irreversible blindness worldwide [1]. Regardless of the type of glaucoma, the most important pathological basis is the persistent death of retinal ganglion cells (RGCs) and their axons, which form the optic nerve [2]. High intraocular pressure (IOP) is the most critical diagnostic and therapeutic target for clinical glaucoma [3, 4]. However, in clinical practice, it has been found that some glaucoma patients still have optic nerve damage even after the IOP has been reduced [5]. Therefore, the optic nerve should be protected while decreasing the IOP.

Gynostemma glycoside, also known as seven-leaf gall, is a perennial herbaceous vine climbing plant of the genus Gynostemma (Gynostemma Blume Bijdr) in the family Cucurbitaceae [6]. It was first recorded in Zhu Nan's “The Materia Medica” in the Ming Dynasty and is known as “the divine herb,” “the herb of immortality and longevity,” “the second ginseng,” and “the southern ginseng.” Gynostemma glycosides have a positive effect on improving microcirculation, scavenging free radicals, as well as improving the nonspecific immunity of the body. It also has anti-inflammatory, antitumor, and antioxidant properties [7, 8]. Gynostemma glycoside has also shown good protective effects in neurological diseases such as Alzheimer's disease, Parkinson's disease, depression, and hypoxic brain injury. Gynostemma glycoside protects nerves through anti-inflammation, antioxidative stress, and promoting nerve regeneration [9]. In this study, we investigated the protective effect of gynostemma glycosides in regulating the STAT3/JAK2 signaling pathway on the optic nerve of rats with chronic high intraocular pressure from the anti-inflammatory aspect so as to identify a safer and more effective drug treatment for patients with glaucomatous optic neuropathy and to further advance research on the use of Chinese medicine for optic nerve protection.

## 2. Materials and Methods

### 2.1. Experimental Subjects

A total of 60 healthy Sprague Dawley (SD) rats of Specific Pathogen Free (SPF) grade (60 males), three-month-old, weighing 180 ± 20 *g*, were supplied by Hunan Shrek Company (certificate of quality no.: 1107272011006979) and fed in the Laboratory Animal Center of Hunan College of Chinese Medicine. All animal studies (including the mice euthanasia procedure) were done in compliance with Hunan University institutional animal care regulations and guidelines and conducted according to the Association for Assessment and Accreditation of Laboratory Animal Care (AAALAC) and the Institutional Animal Care and Use Committee (IACUC) guidelines. There was no obvious abnormality in the anterior segment and fundus examination.

### 2.2. Experimental Drugs

Gynostemma glycosides were provided by the Shaanxi Guanjie Biological Technology Co., Ltd (quality points ≥ 98%; batch no. GY20200323).

### 2.3. Reagents and Experimental Equipment

Reagents were rabbit secondary antibody (CoraLite594-conjugated Goat Anti- Rabbit IgG (*H* + *L*), Proteintech, Rosemont, IL, USA, article number SA00013-4), rabbit secondary antibody (CoraLite594-conjugated Donkey IgG (*H* + *L*), Proteintech, Rosemont, IL, USA, article number SA00013-8), goat secondary antibody (Fluorescein (FITC)-conjugated Affinipure Donkey Anti-Goat IgG (*H* + *L*), Proteintech, Rosemont, IL, USA, article number SA00003-3), mouse secondary antibody (horseradish peroxidase (HRP)-conjugated AffiniPure Goat Anti-Mouse IgG (*H* + *L*) Proteintech, Rosemont, IL, USA, article number SA00001-1), and rabbit secondary antibody (HRP-conjugated AffiniPure Goat Anti-Rabbit IgG (*H* + *L*), Proteintech, Rosemont, IL, USA, article number SA00001-2).

Instruments included an inverted microscope (Motic, Wetzlar, Germany), fluorescence microscope, MDF-382E ultralow temperature refrigerator (Sanyo, Osaka, Japan), TONO-Pen AVIA tonometer (Medtronic SALON, USA), and HE staining kit (Bioswamp).

### 2.4. Modeling and Grouping

Referring to the previously published method [10], we cauterized the superficial scleral vein to establish a chronic high intraocular pressure model. Under the microscope, a radial incision is made 2 mm from the corneal limbus to cut the lateral and superior bulbar conjunctiva; carefully separating the fascia and muscles; exposing 2 or 3 suprascleral veins in the superior nasal, superior temporal, and inferior temporal quadrants; and then cauterizing these 3 suprascleral veins with an ophthalmic surgical hemostat until the venous flow disappears and the proximal veins are filled with blood and rage. Ten out of the 60 rats were randomly selected as group A (the blank group), and the remaining 50 rats were used to establish the chronic hypertensive model. The IOP was measured before, at 30 min, 7 d, and 14 d after modeling. Rats with a mean IOP above 22 mmHg (1 mmHg = 0.133 kPa) were considered for the next experiment. A second modeling session was performed if the postoperative IOP was not increased or if it increased and then decreased. If the second modeling was also unsuccessful, the failed rats were excluded from the study. Fifty rats with IOP above 22 mmHg were randomly divided into group B: negative control group; group C: gynostemma low-dose group; group D: gynostemma medium-dose group; group E: gynostemma high-dose group; and group F: positive control group. A total of 5 ml of saline gavage was used for group B; 25, 50, 100 mg/(kg/d) of gynostemma gavage in groups C, D, and F, respectively; 5 ml of VitB1 and VitB12 gavage in group E. VitB12 was administrated by gavage. All groups were daily gavaged in the early morning for 14 days and treated with 0.5% timolol eye drops twice a day to control the intraocular pressure during the treatment period. In our experiments, we used the Tono-pen IOP agent to measure IOP in rats. This IOP meter works by continuous contact with the cornea to obtain IOP values, and its IOP measurement results are not affected by the hardness of the eye wall, so its IOP measurement values are more accurate. The mean value was recorded after local anesthesia in the right eye of rats.

### 2.5. Sampling Method

Their eyeballs were removed under general anesthesia after two-week gavage. The anterior segment of the eye and vitreous was removed under a microscope, and the retinal tissue was peeled out with microforceps. One piece of the tissue was used to preserve 4% paraformaldehyde, conventional paraffin embedding, and serial sections for immunohistochemical assays; the other piece was frozen and preserved for RT-PCR assays.

### 2.6. Histopathological Observation

All rats were killed through air embolism. After that, we performed enucleation procedures on these rats. The operation sites of enucleated eyes were dissected into blocks that contained retinal tissue and optic nerve. After that, we performed HE staining and LFB staining to detect the number of CD11b (the goat anti-human primary antibodies (1 : 50), ThermoFisher), GFAP (the rabbit anti-human primary antibodies (1 : 50), PTG), Brn3*α* (the rabbit anti-human primary antibodies (1 : 50), Abcam), and TUNEL content. To determine Brn3*α* and TUNEL content, the slices were immersed in citrate buffer (pH6.0) and heated to boiling in an electric furnace or microwave oven, after which they were cut off after boiling for 23 min, cooled for 23 min, and then removed and cooled to room temperature. Then, 0.01 M PBS (pH 7.2∼7.6) was used for washing 3 times after cooling, after which appropriate antibodies were added. DAPI working solution was used to stain the nuclei at 37°C for 10 min, and after buffered glycerol sealing, the slices were observed under a fluorescence microscope (magnification of 40x and 10x).

### 2.7. Quantitative RT-PCR

After performing scleral vein cauterization on the eyes of rats, we harvested their tissues, including retinal tissue and optic nerve, on postoperative day 14 (D14). The total RNA was extracted from the tissues using Trizol (Thermo, the United States). An ultraviolet spectrophotometer (Thermo, the United States) was then used to quantify and examine the quality of the isolated RNAs. 5 µg of total RNA was then reversely transcribed in cDNAs using quantitative RT-PCR. The DDCT method (2^−△△Ct^) was applied to calculate the relative differences between the model group and treatment groups, and the results were expressed as fold changes in gene expression. The forward and reverse primers were as follows: R-actin, F ACATCCGTAAAGACCTCTATGCC, R TACTCCTGCTTGCTGATCCAC, product length 223bp; R-STAT3, F ATGTCCTCTATCAGCACAACC, R GACTCTTCCCACAGGCATCGG, product length 112bp; R-JAK2, F TACTTCCTGACCTTTGCCGTTG, R AGGTTTGATTTATCTTTCGGCTT, product length 224bp.

### 2.8. Western Blot

Samples of retinal tissue and optic nerve were subjected to radioimmunoprecipitation assay buffer. First is the sodium laurylsulfate. The polyacrylamide gel electrophoresis method was used for separating proteins of different molecular weights and then transferring them onto polyvinylidene difluoride membranes. After the end of the transformation of the membranes, the membranes were blocked, and the rabbit anti-human primary antibodies (1:2000) of STAT3, p-JAK2 proteins, the rabbit anti-human primary antibodies (1∶3000) of p-STAT3 proteins, and the rabbit anti-human primary antibodies (1:750) of JAK2 proteins were incubated according to the relative molecular mass of the marker, and the HRP-labeled anti-rabbit IgG secondary antibody (dilution, 1:5000) was used. The film is incubated with ECL chemiluminescent solution, plasticized and developed and rinsed in a dark box with X-film exposure for 1–60 minutes.

### 2.9. HE Staining

The sections were incubated in xylene for 15 min, 3 times, after which they were sequentially placed in 100%, 100%, 95%, 85%, and 75% ethanol (5 min for each step). Samples were then washed with distilled water for 5 minutes and dehydrated in gradient alcohol (95–100%) (5 min for each step). After being removed and placed in xylene for 10 min, neutral gum sealing and microscopic observation were performed 2 times.

### 2.10. Statistical Analysis

The data were statistically analyzed using SPPS 22.0 software (IBM, Armonk, NY, USA), and the measured data were expressed as mean ± standard deviation ($\bar{x}$ ± s). The single-factor ANOVA was used for making a comparison between the metrological data in accordance with normal distribution and variance homogeneity, and the pair-wise comparisons between multiple groups were performed with Student's *t*-test. *P* < 0.05 indicated that the difference was significant, and *P* < 0.01 indicated that the difference was extremely significant.

## 3. Results

### 3.1. Intraocular Pressure Measurement Results

Before modeling, there was no statistical significance in the IOP of the 6 groups. 30 min after modeling, the IOP of groups B, C, D, E, and F increased compared with before, and modeling was successful. At 1 and 2 weeks after modeling, IOP in groups B, C, D, E, and F was higher than that in group A. After modeling, the IOP of groups B, C, D, E, and F was not statistically significant (Table 1).

### 3.2. HE Staining

The structure of the retinal layers in group A was clear, and the cells in each layer were arranged in a regular and orderly manner. The remaining five groups showed thinning of retinal structure, retinal edema, irregular arrangement and disorderly distribution of RGCs, reduced number of cells, and formation of vacuoles. However, the arrangement of RGCs in groups C, D, and E was more regular than that in groups B and F. The number of RGCs in the gynostemma glycosides high-dose group was mildly reduced, and a small number of vacuoles were formed. In groups D and E, the structure of the retinal layers was clear, the RGCs were neatly and densely arranged, and the edema significantly improved (Figure 1).

### 3.3. Brn3*α*-TUNEL Staining

Regarding TUNEL and Brn3*α* expression, normal retinal tissues had no obvious green-red granules in the cytoplasm. Group A showed few granules, indicating that TUNEL cells and Brn3*α* were not clearly expressed. Many particles appeared in group B, and fewer green-red particles appeared after treatment with gynostemma glycosides suggesting negative expression of TUNEL cells and Brn3*α*. At all time points, only a few green-red particles appeared in group E, which roughly resembled those in group A (Figure 2 and Table 2).

### 3.4. CD11b-GFAP Staining

Regarding GFAF and CD11b, normal retinal tissues had no obvious green-red granules in the cytoplasm. Group A showed few granules, indicating that GFAF and CD11b were not clearly expressed. However, many particles appeared in group B, and fewer green-red particles appeared after treatment with gynostemma glycosides, suggesting negative expression of TUNEL and Brn3*α*. At any given time, only a few green-red particles appeared in group E, which roughly resembled those in group A (Figure 3 and Table 3).

### 3.5. qRT-PCR Detection of STAT3 and JAK2 mRNA Expression

Reverse transcription PCR showed that the relative expression of STAT3 and JAK2 mRNA in the gynostemma glycosides treatment groups was significantly lower compared to group B (*P* < 0.05). In groups D and E, these expressions were significantly lower than those in group F (*P* < 0.05), while group E had lower expressions than those in group D (*P* < 0.05) (Figure 4 and Table 4).

### 3.6. Western Blot

The expression of STAT3 and JAK2 in groups A, C, D, E, and F was significantly lower than in group B (*P* < 0.05). Moreover, the expression of STAT3 and JAK2 in groups D, and E was lower than in group F (*P* < 0.05), and the expression of STAT3 and JAK2 in group E was lower than in group D (*P* < 0.05) (Figure 5 and Table 5).

## 4. Discussion

Glaucoma is a degenerative disease of CNS neurons that shares some similar neurobiological features with Alzheimer's disease (AD)/Parkinson's disease (PD)/multiple sclerosis (MS); however, the pathogenesis of the disease may differ in terms of the anatomical localization of the damaged nucleus accumbens and the unique initiation mechanism [11]. Retinal ganglion cells (RGCs) are directly exposed to a variety of specialized immune cells such as microglia (which can activate and mediate the immune-inflammatory response), astrocytes, and Muller cells, capillaries. Increased activity of these immune cells can lead to alterations in the blood-retinal barrier and, in turn, affect the environment in which RGCs/axons survive, leading to glaucoma [12–16].

In addition to their immune cell-like role, astrocytes build the integrity of the blood-brain barrier and the blood-retinal barrier. Studies of other central neurodegenerative pathologies, including AD and PD, have found that prolonged activation of microglia and release of a range of inflammatory factors can cause neuronal damage [17, 18]. After activating the astroglial fine run, cytokines, chemokines, and complement components may be upregulated, disrupting the barrier integrity. Consequently, peripheral immune cells may enter the central nervous system (CNS) through the disrupted barrier and participate in the neuroimmune inflammatory processes, accelerating neuronal loss [19, 20]. Thus, we hypothesized that the mechanism through which gibberellin protects RGCs might also be related to the neuroimmune inflammatory response [21, 22]. We hypothesized that STAT3/JAK2, a major intracellular signaling pathway, is associated with the astrocyte activation process.

When apoptosis occurred in the retinal tissue, the extent of apoptosis in RGCs could be studied by Brn3*α*-TUNEL staining. After 14 d of treatment with high-dose gibberellin saponin, the number of TUNEL-Brn3*α*-positive cells was reduced compared with the negative control group (*P* < 0.01), which indicated that high-dose gibberellin saponin exerted a protective effect against persistent apoptosis of retinal RGCs caused by chronic high IOP.

The amount of microglia and astrocytes in the optic nerve is reflected by the expression of CD11b and GFAP detected by immunostaining. The expression of both of these biomarkers was significantly reduced in all groups treated with gynostemma saponin (*P* < 0.05), and the best inhibition was observed in the high-dose group (*P* < 0.05). These results suggest that gynostemma saponin can effectively inhibit the expression of inflammatory microglia and astrocytes in the retina and slow down the development of retinal inflammation in the rat model of chronic high IOP.

STAT3/JAK2 is expressed in retinal astrocytes and is a major intracellular signaling pathway during astrocyte activation [23, 24]. Astrocytes are activated early after an acute hypertensive eye injury. The intracellular STAT3/JAK2 signaling pathway appears to be activated in glial cells at an early stage, with retinal ganglion cells showing more obvious damage after glial cell activation [25, 26]. After optic nerve injury, the microenvironment in which RGCs survive can be altered, inducing secondary apoptosis of RGCs, that can cause irreversible loss of vision [27–29]. In this study, we found that gypenoside can inhibit the amplification of STAT3 mRNA and JAK2 mRNA in the retina, thereby inhibiting the activation of glial cells and neuroimmune inflammation. The results of HE staining indicated that, in the high-dose gypenoside treatment group, the structure of each layer of the retina was clear, the RGCs were neatly and densely arranged, and the retinal edema was significantly improved compared with the negative control group, which indicated that gypenosides could inhibit STAT3 mRNA and JAK2 mRNA and further protect RGCs. Among these groups, the best effect was observed in the high-dose group.

Chinese medicine has been used for decades to improve and prevent symptoms of hypertension, bronchial dilation, diabetes, myocardial infarction, bronchitis, hepatitis, and hypogonadism [7, 8, 30, 31]. Our previous studies demonstrated that gynostemma glycosides have antitumor, antioxidant, and anti-inflammatory properties and can inhibit the expression of inflammatory factors, retinal protective effects, and activation of proinflammatory enzymes [32–35].

In this paper, we further investigated the anti-inflammatory effect of gynostemma based on the regulation of the STAT3/JAK2 signaling pathway. During the development of glaucoma, the microenvironment at the optic disc activates glial cells, causing them to release inflammatory factors and trigger immune responses. Moreover, some inflammatory factors could further affect the function of glial cells and RGCs. The inflammatory and immune responses caused by glial cell activation can lead to the death of retinal RGCs and sieve plate remodeling and optic disc damage. Activation of astrocytes and microglia at the optic disc site is seen in the early stage of glaucoma, and microglia affects apoptosis of RGCs through altered morphology, genetics, cell proliferation, and immune response throughout the pathogenesis of glaucoma. Therefore, optic nerve protection is achieved through anti-inflammation during the pathogenesis of glaucoma.

In this study, we confirmed that gibberellin saponin inhibits the amplification of STAT3 mRNA and JAK2 mRNA in the retina, downregulates STAT3 and JAK2, and suppresses the activation of astrocytes and microglia. These data are expected to help identify a safer and more effective pharmacological treatment for patients with glaucomatous optic neuropathy in clinical practice and open up new fields for further research on optic nerve protection in Chinese medicine.

The main limitation of the present study is failing to determine which gene locus was the malefactor at the genetic level. The pathway blockers should be applied to block the pathway loci one by one to confirm the reliability of the pathway, which is the direction of our further research. Another important issue is the prevention of RGCs. There are many methods to prevent apoptosis, such as gene regulation, microenvironmental changes, and hepatocyte transplantation, which have been experimentally studied and shown to be effective. However, all of these are limited to the basic research stage and lack practical clinical significance.

To sum up, our study showed that gynostemma glycosides are clinically effective in treating optic nerve damage caused by optic neuritis. Thus, gynostemma glycosides should be considered as an effective drug candidate for optic nerve injury.

## Figures and Tables

**Figure 1:** Observation of the retinal structure of each group by HE staining (light microscope 400x). (a) The blank group; (b) negative control group; (c) gynostemma glycosides low-dose group; (d) gynostemma glycosides medium-dose group; (e) gynostemma glycosides high-dose group; (f) positive control group.

**Figure 2:** Immunohistochemical staining of Brn3*α*-TUNEL (light microscope 400×). (a) the blank group; (b) negative control group; (c) gynostemma glycosides low-dose group; (d) gynostemma glycosides medium-dose group; (e) gynostemma glycosides high-dose group; (f) positive control group.

**Figure 3:** Immunohistochemical staining of CD11b (DAPI staining and GFAP immunofluorescence staining, light microscope 400x). (a) The blank group; (b) negative control group; (c) gynostemma glycosides low-dose group; (d) gynostemma glycosides medium-dose group; (e) gynostemma glycosides high-dose group; (f) positive control group.

**Figure 4:** Relative expression of STAT3 and JAK2 mRNA. (a) The blank group; (b) negative control group; (c) gynostemma glycosides low-dose group; (d) gynostemma glycosides medium-dose group; (e) gynostemma glycosides high-dose group; (f) positive control group.

**Figure 5:** Electrophoresis diagrams of JAK2, P-JAK2, STAT3, and P-STAT3 protein expression of rats by western blot in each group. (a) The blank group; (b) negative group; (c) gynostemma glycosides low-dose group; (d) gynostemma glycosides medium-dose group; (e) gynostemma glycosides high-dose group; (f) positive control group.

**Table 1:** Comparison of IOP before and after modeling in each group of rats (mean ± SD, *n* = 10).

Group	IOP (mmHg)			
	Before molding	30 minutes after mold making	1 week after mold making	2 weeks after mold making
A	13.43 ± 0.99	13.34 ± 0.74	13.78 ± 0.74	14.05 ± 1.06
B	13.30 ± 0.86	32.04 ± 4.42^ab^	31.86 ± 4.42^ab^	33.53 ± 3.20^ab^
C	13.30 ± 0.82	34.42 ± 4.94^ab^	30.57 ± 4.94^ab^	35.71 ± 2.61^ab^
D	13.30 ± 0.90	34.46 ± 3.17^ab^	31.72 ± 3.17^ab^	36.64 ± 2.64^ab^
E	13.54 ± 0.90	33.12 ± 4.44^ab^	32.61 ± 4.44^ab^	36.09 ± 2.68^ab^
F	13.30 ± 0.94	32.01 ± 3.45^ab^	31.77 ± 3.35^ab^	32.19 ± 2.42^ab^

Notes: A: the blank group; B: negative control group; C: gynostemma glycosides low-dose group; D: gynostemma glycosides medium-dose group; E: gynostemma glycosides high-dose group; F: positive control group. Compared with group A, ^a^*P* < 0.05. Comparison with the same group before modeling, ^b^*P* < 0.05.

**Table 2:** Comparison of the mean fluorescence intensity value in each group (mean ± SD, *n* = 10).

Group	Brn3*α*	TUNEL
A	0.005 ± 0.002^a^	0.005 ± 0.003^a^
B	0.188 ± 0.225	0.143 ± 0.006
C	0.761 ± 0.173^ab^	0.419 ± 0.008^a^
D	0.565 ± 0.045^a^	0.457 ± 0.009^a^
E	0.012 ± 0.014^ab^	0.017 ± 0.027^ac^
F	0.389 ± 0.058^a^	0.041 ± 0.005^a^

Notes: A: the blank group; B: negative control group; C: gynostemma glycosides low-dose group; D: gynostemma glycosides medium-dose group; E: gynostemma glycosides high-dose group; F: positive control group. Compared with group B, ^a^*P* < 0.05. Compared with group F, ^b^*P* < 0.05. Compared with group F, ^c^*P* < 0.05.

**Table 3:** Comparison of the mean fluorescence intensity value in each group (mean ± SD, *n* = 10).

Group	GFAP	CD11b
A	2598.75 ± 817.0^a^	10605.00 ± 2077.51^a^
B	105445.75 ± 7473.45	220883.00 ± 20127.62
C	26169.25 ± 3696.26^a^	129973.50 ± 10002.24^a^
D	15195.25 ± 3676.64^a^	123341.75 ± 13022.53^a^
E	7990.25 ± 1058.92^ab^	86239.75 ± 15253.32^ab^
F	20608.50 ± 2143.46^a^	126671.50 ± 19693.70^a^

Notes: A: the blank group; B: negative control group; C: gynostemma glycosides low-dose group; D: gynostemma glycosides medium-dose group; E: gynostemma glycosides high-dose group; F: positive control group. Compared with group B, ^a^*P* < 0.05. Compared with group F, ^b^*P* < 0.05.

**Table 4:** Relative expression of STAT3 and JAK2 mRNA (mean ± SD, *n* = 10).

Group	STAT3 mRNA	JAK2 mRNA
A	0.91 ± 0.13^a^	0.93 ± 0.11^a^
B	6.65 ± 0.88	7.89 ± 0.35
C	4.66 ± 0.53^a^	5.62 ± 0.71^a^
D	3.15 ± 0.18^ab^	3.26 ± 0.23^ab^
E	1.71 ± 0.09^abc^	1.88 ± 0.19^abc^
F	4.67 ± 0.32^a^	5.69 ± 0.77^a^

Notes: A: the blank group; B: negative control group; C: gynostemma glycosides low-dose group; D: gynostemma glycosides medium-dose group; E: gynostemma glycosides high-dose group; F: positive control group. Compared with group B, ^a^*P* < 0.05. Compared with group F, ^b^*P* < 0.05. Compared with group D, ^c^*P* < 0.05.

**Table 5:** Electrophoresis diagrams of JAK2, P-JAK2, STAT3, and P-STAT3 protein expression of rats in each group (mean ± SD, *n* = 10).

Group	STAT3	JAK2	P-STAT3	P-JAK2
A	0.91 ± 0.11^a^	0.93 ± 0.11^a^	3.45 ± 2.38^a^	12.61 ± 3.42^a^
B	6.65 ± 0.88	7.89 ± 0.35	36.15 ± 4.91	40.76 ± 4.93
C	4.66 ± 0.53^a^	5.62 ± 0.71^a^	31.13 ± 3.48^a^	33.29 ± 5.79^a^
D	3.15 ± 0.18^ab^	3.26 ± 0.23^ab^	24.54 ± 4.36^ab^	28.39 ± 7.56^a^
E	1.71 ± 0.09^abc^	1.88 ± 0.19^abc^	15.62 ± 6.12^abc^	24.49 ± 8.49^a^
F	4.67 ± 0.32^a^	5.69 ± 0.77^a^	33.73 ± 5.42^a^	35.39 ± 6.12^a^

Notes: A: the blank group; B: negative control group; C: gynostemma glycosides low-dose group; D: gynostemma glycosides medium-dose group; E: gynostemma glycosides high-dose group; F: positive control group. Compared with group B, ^a^*P* < 0.05. Compared with group F, ^b^*P* < 0.05. Compared with group D, ^c^*P* < 0.05.

## Data Availability

The data used to support the findings of this study are included within the article.

## Additional Points

*Synopsis.* Gynostemma glycosides had a protective effect on retinal ganglion cells in rats with chronic high intraocular pressure, and the effect of high doses of gynostemma glycosides was optimal.
